# Belinostat and panobinostat (HDACI): in vitro and in vivo studies in thyroid cancer

**DOI:** 10.1007/s00432-013-1465-6

**Published:** 2013-07-04

**Authors:** Daniel Chan, Yun Zheng, Jeffrey W. Tyner, Wee Joo Chng, Wen Wen Chien, Sigal Gery, Geraldine Leong, Glenn D. Braunstein, H. Phillip Koeffler

**Affiliations:** 1 National University Hospital, National University Cancer Institute Singapore, 1E Kent Ridge Road, Singapore, 119228 Singapore; 2 Division of Hematology/Oncology, Cedars-Sinai Medical Center, University of California at Los Angeles School of Medicine, 8700 Beverly Boulevard, Los Angeles, CA 90048 USA; 3 Oregon Health and Science University, 3181 S.W. Sam Jackson Park Rd., Portland, OR 97239-3098 USA; 4 Cancer Science Institute Singapore, Centre for Translational Medicine, NUS, 14 Medical Drive, MD6, #12-01, Singapore, 117599 Singapore; 5 State Key Laboratory of Oncology in South China, Cancer Center, Sun Yat-sen University, 651 Dongfeng East Rd, Guangzhou, 510060 People’s Republic of China

**Keywords:** Histone deacetylases, Tyrosine kinase inhibitors, Thyroid cancer, Novel therapeutic approach

## Abstract

**Purpose:**

Advanced thyroid cancer responds poorly to most therapies. New therapies and combinations are needed. The aim of this study was to examine both in vitro and in vivo activity of two relatively new histone deacetylase inhibitors (HDACIs), belinostat and panobinostat, and a variety of tyrosine kinase inhibitors (TKIs) against a panel of nine human thyroid cancer cell lines.

**Methods:**

The anti-proliferative activity and the effects of HDACIs, TKIs and their combinations on thyroid cancer cells were determined by cytotoxicity assays, microarray and immunoblot analyses. Synergism between HDACIs and TKIs was assessed by the median effects model of Chou-Talalay (Calcusyn^®^).

**Results:**

Belinostat and panobinostat were active against the thyroid cancer cell lines irrespective of their mutational composition, and belinostat was effective in preventing growth of human thyroid cancer xenografts in immunodeficient mice. Further studies showed that both HDACIs induced apoptosis. HDACI also elevated acetylated histone 3, p21^Waf^, and PARP, and decreased levels of phosphorylated ERK and AKT (Ser473). RNA assay analysis suggested both HDACIs modulated genes associated with the cell cycle, DNA damage and apoptosis. Most of the TKI (pazopanib, motesanib, sorafenib and dasatinib) were either inactive in vitro or were active only at high doses. However, the novel combinations of either pazopanib or dasatinib TKIs with either belinostat or panobinostat synergistically inhibited cell growth of thyroid cancer cells in vitro.

**Conclusions:**

In summary, these HDACIs either alone or combined with selected TKIs may have a role in treatment of aggressive thyroid cancer.

**Electronic supplementary material:**

The online version of this article (doi:10.1007/s00432-013-1465-6) contains supplementary material, which is available to authorized users.

## Introduction

Therapies for metastatic advanced thyroid cancers are inadequate with most therapeutic approaches failing to produce meaningful long-term responses (Smallridge et al. 2009; Licitra et al. 2010). The relatively modest response rates with tyrosine kinase inhibitors (TKIs) have led to several ongoing trials using combinations of TKIs with other targeted agents in an effort to improve the clinical outcome (Cohen et al. 2008; Gupta-Abramson et al. 2008; Sherman et al. 2008; Schlumberger et al. 2009; Bible et al. 2010).

Histone deacetylase inhibitors (HDACIs) are a promising class of drugs in thyroid cancer; in vitro and in vivo studies of vorinostat (SAHA) (Luong et al. 2006) showed that this agent is active against human thyroid cancer cell lines. However, data suggest that single-agent HDACIs may not be a viable treatment strategy in solid cancers (Ellis and Pili 2010; Woyach et al. 2009; Venugopal and Evans 2011). As such, a number of trials are pursuing combinations of HDACIs with other agents both in thyroid cancer and other types of solid malignancies (Munster et al. 2011). In this study, we tested two relatively new HDACIs (belinostat and panobinostat) and multiple TKIs alone and in combination against a panel of nine human thyroid cancer cell lines that have been validated as to their accuracy (Schweppe et al. 2008); these HDACIs appear active both in vitro and in vivo (belinostat) and appear to have enhanced activity when combined with one of several TKIs.

## Materials and methods

### Reagents

Belinostat and panobinostat (HDACIs) were obtained from National Cancer Institute (NCI, USA) and Selleck Chemicals (Boston, MA), respectively. Pazopanib, motesanib, sorafenib and dasatinib (TKIs) (LC Laboratories) were dissolved in DMSO and stored in aliquots at −20 °C until use. Antibodies to acetylated histone H3 (AcH3), p21^Waf1^, PARP, pAKT (Ser473), pERK, AKT, ERK and GAPDH were obtained from Cell Signaling Technology (MA, USA).

### Cell lines and culture

Cal62 (anaplastic—KRAS G12R mutant), SW1736 (anaplastic—BRAF mutant), T238 (anaplastic—PI3K and BRAF mutant), Hth7 (anaplastic—NRAS Q61R), T241 (unknown—no mutation), T351 (unknown—no mutation), C643 (anaplastic—HRAS G13R), BHP2-7 (papillary—RET/PTC rearrangements) and Hth83 (unknown—HRAS G13R) were generously provided by Dr. James A. Fagin (Memorial Sloan Kettering Cancer Center, New York, USA). Hth7 was grown in DMEM with 10 % fetal bovine serum (Hyclone, Logan, UT). The rests of the cell lines were maintained in RPMI (Life Technologies, Carlsbad, CA) containing 10 % fetal bovine serum, 1 % penicillin–streptomycin and 1 % glutamine with the exception of SW1736, which was supplemented with 1 % MEM non-essential amino acid. All cells were grown at 37 °C and 5 % CO_2_.

### Cytotoxicity assay

For measurement of cell viability, 1.0–5.0 × 10^3^ cells were plated in 96-well flat-bottomed microtiter plates and grown overnight at 37 °C. The following day, the cells were treated with 10 μl of various concentrations of either HDAC inhibitors/TKI/combination or vehicle and incubated for 48/72 h. After 48/72 h, 250 μg of MTT [3-(4,5-dimethylthiazol-2-yl)-2,5-diphenyltetrazolium bromide] (Sigma-Aldrich) was added to each well and incubated at 37 °C for 2–4 h, after which 100 μl of DMSO was added, as previously reported (Chan et al. 2012). Absorbance was measured with a Tecan Infinite 200 PRO spectrophotometer (Mannedorf, Switzerland) at a wavelength of 595 nm. As previously mentioned, the percentage viability at each drug concentration was calculated using the following formula:

$$ \frac{{({\text{Absorbance}}\;{\text{of}}\;{\text{treated}}\;{\text{cells}} - {\text{Absorbance}}\;{\text{of}}\;{\text{media}})}}{{({\text{Absorbance}}\;{\text{of}}\;{\text{untreated}}\;{\text{cells}} - {\text{Absorbance}}\;{\text{of}}\;{\text{media}})}} $$

The percentage values obtained were then plotted using GraphPad Prism^®^ software nonlinear regression (curve fit) to obtain the half maximal inhibitory concentration (IC_50_) and its 95 % confidence interval (CI).

The dose ranges tested: belinostat (100–10,000 nM); panobinostat (1–2,000 nM); dasatinib (1–300 nM); sorafenib, pazopanib and motesanib (100–5,000 nM).

### Assessment of synergism by the median effects model of Chou-Talalay (Calcusyn^®^)

The combinations of HDACIs and TKIs were assessed by the median effects model of Chou-Talalay using Calcusyn^®^ software from BioSoft^®^. The interpretation of the normalized isobolograms and interpretation of the degree of synergism is as per the combination index (CI) stated in Supporting Information Fig. S1.

### Gene expression profiling and analysis

Using Affymetrix Human Gene 1.0ST array (Affymetrix, Santa Clara, CA), mRNA expression profiling was done in either biological triplicates (for BHP control and BHP panobinostat 100 nM, 30 h) or biological duplicates (BHP belinostat 50 μM, 30 h). Total RNA was reversed transcribed, amplified and labeled according to manufacturer’s protocol. Labeled cDNA was hybridized onto Human Gene 1.0ST array for 16 h at 60 rpm in a GeneChip Hybridization Oven 640 (Affymetrix). Following manufacturer’s instructions, the arrays were washed and scanned using GeneChip Scanner 3000 7G. The CEL files were imported into GeneSpring Software V11 for data normalization and identification of differentially expressed mRNAs of interest. As mentioned previously, the CEL files were preprocessed using RMA16 algorithm and CORE transcript level. Data were quantile normalized, and those expression values less than the 20th percentile were filtered out. A list of differentially expressed mRNAs of interest was generated using the fold change function (Chan et al. 2012). Using hierarchical clustering, heatmaps were generated and gene ontology analysis was done using GO. To understand further the biological functions of the differentially expressed genes, Web-based software, MetaCore (GeneGo, St. Joseph, MI), was used to perform gene ontology and pathway/network analysis as mentioned previously (Chan et al. 2012). Several algorithms to enable both the construction and analysis of gene networks were integrated as previously described (Ekins et al. 2007).

### Western blotting

Lysates were collected from cells treated with HDAC inhibitor for 30 h. Briefly, cells were lysed at 4 °C in RIPA lysis buffer, and the insoluble material was removed by centrifugation at 4 °C, 10,000*g* for 10 min. Proteins in the cell lysates were quantified by Bradford Assay. Forty micrograms of protein from each sample was resolved by SDS-PAGE and electroblotted to Immobilon-P Transfer Membranes (Millipore, Billerica, MA). Membranes were probed with the various primary antibodies from Cell Signaling Technologies. Following binding of the primary antibodies, horseradish peroxidase (HRP)-conjugated anti-rabbit/anti-mouse secondary antibodies were introduced to the membrane. Bound secondary antibody was detected by using Amersham ECL Plus Western blotting detection reagents (GE Healthcare, USA). Membranes were stripped and probed for GAPDH as loading controls or the non-phosphorylated protein (where applicable) (Chan et al. 2012).

### Apoptosis assay

According to the instructions from the manufacturer, 10^5^ cells were treated with either belinostat or panobinostat for 48 h and labeled with FITC-conjugated annexin V antibody and propidium iodide (PI) using annexin V–FITC Apoptosis Detection kit I (BD Biosciences, San Jose). Positive cells were detected by fluorescence-activated cell sorting as mentioned previously (Chan et al. 2012).

### Murine studies

All mice were fed a standard chow diet. Six-week-old female athymic nu/nu mice—NCRFU—were purchased from Taconic Hudson (NY). Upon arrival, these animals were quarantined for 1 week in the animal facility and maintained in a 12 h light/dark cycle, with free access to food and water.

Mice were anaesthetized with inhalational isoflurane (Hospira Lakeforest, IL). BHP2-7 cells (2 × 10^7^) were resuspended in 50 μl Matrigel (BD Biosciences) and 50 μl PBS for each tumor. Cells were injected subcutaneously on both flanks of the immunodeficient mice. A total of 32 tumors were inoculated (8 in control and 8 in drug treatment mice). Mice were injected with belinostat intraperitoneal (Cheung et al. 2003) (100 mg/kg/injection), 5 days a week for 3 weeks starting on day 3. The weight of the mice was measured every week. At the end of either drug or vehicle-only treatment (52 days after tumor cell injection), animals were killed by CO_2_ inhalation, tumor dissected and volumes calculated according to the formula: (length × width × thickness × 0.5236) (Chan et al. 2012). During the experiment, external measurements were made in millimeters using vernier callipers. At completion of the study, tumors were formalin-fixed and processed for histological and immunohistochemical (IHC) analyses. Murine studies were approved by the Animal Care and Use Committee of Cedars-Sinai Medical Center, and all animal care was in accordance with the IACUC guidelines.

## Results

### Cytotoxicity assay

To assess the anti-proliferative activity of either the HDACIs or TKIs, dose–response studies were performed using MTT assay. Mean proportion viability of the cells at each drug concentration was plotted using GraphPad Prism software^®^, and the drug dose that inhibited 50 % growth (relative to vehicle-treated control) [IC_50_] at 72 h of culture was obtained from the software (nonlinear regression curve fit). For range of drug testing, the pharmacologically relevant doses of each of the drugs were inferred from phase I clinical trials (see “Materials and methods”) (Giles et al. 2006; Hurwitz et al. 2009; Minami et al. 2008; Demetri et al. 2009; Schlumberger et al. 2009; Steele et al. 2008). Both belinostat and panobinostat reduced thyroid cancer cell viability in vitro in 8 of the 9 cell lines tested at a pharmacologically achievable dose; the PI3K + BRAF mutant (T238) cell line was resistant to panobinostat (Table 1). Only sorafenib [8 of 9 cell lines (IC_50_ 5.0–13 μM)], pazopanib [1 of 9 cell lines (IC_50_ 3.4 ± 0.2 μM)] and dasatinib [2 of 9 cell lines, (IC_50_ 47 ± 3 and 35 ± 5 nM)] were effective among the TKIs (Table 1).

**Table 1:** Dose of drug that inhibited 50 % growth of human thyroid cancer cell line in vitro

Cell line	Mutation/arrangements	IC50 (nM) Belinostat	IC50 (nM) Panobinostat	IC50 (nM) Dasatinib	IC50 (μM) Sorafenib	IC50 (nM) Pazopanib	IC50 Motesanib
Cal62	KRAS	470 ± 36	33 ± 4	35 ± 5	13 ± 1.1	NR	NR
Hth7	NRAS	400 ± 56	15 ± 2	NR	6.8 ± 0.8	NR	NR
Hth83	HRAS	720 ± 100	34 ± 5	NR	11 ± 1.0	NR	NR
C643	HRAS	970 ± 120	71 ± 10	NR	6.5 ± 0.9	NR	NR
SW1736	BRAF	380 ± 40	35 ± 8	NR	NR	NR	NR
T241	Nil	750 ± 65	65 ± 7	NR	7.5 ± 0.5	NR	NR
T351	Nil	1,100 ± 170	50 ± 10	NR	11 ± 2.0	NR	NR
BHP2-7	RET/PTC	770 ± 67	37 ± 6	47 ± 3	5.0 ± 0.8	340 ± 20	NR
T238	PI3 K/BRAF	6,800 ± 740	1,500 ± 200	NR	6.5 ± 1.2	NR	NR

Tabulated results of HDACI (belinostat and panobinostat) and tyrosine kinase inhibitor (TKI dasatinib, sorafenib, pazopanib and motesanib)-treated thyroid cancer cell lines at 72 h of drug exposure. Mean 50 % inhibitory concentration (IC50 ± SD) of experiments done in triplicate experiments with each experiment done with triplicate wells using MTT assay. Nil: No mutations detected. NR: IC50 not reached (i.e., pharmacologically relevant IC50 not reached). See “Materials and methods” for details

### Belinostat- and panobinostat-treated BHP2-7 thyroid cancer cell line has overlapping mRNA changes

In order to gain insights into which common pathways is altered by the two HDACIs, BHP2-7 cells were exposed to either belinostat 50 μM or panobinostat 100 nM for 30 h. RNA was extracted and subjected to microarray analysis (Supporting Information Table S1). Only genes with ≥twofold change (panobinostat treatment) or ≥fourfold change (belinostat treatment) were deemed to be significantly altered. Among the 528 and 573 altered genes for panobinostat and for belinostat, respectively, 153 of these genes were commonly altered. These 153 genes constituted 3 main pathways: cell cycle-related, DNA damage and apoptosis (Supporting Information Fig. S2) which prompted additional studies.

### Belinostat and panobinostat treatment-related protein changes

Both belinostat and panobinostat caused acetylation of histone H3 and induced the expression of p21^Waf1^ in four representative thyroid cancer cell lines (Cal62, SW1736, T238 and BHP2-7) irrespective of their mutational composition (Fig. 1, Panel a). Of note, T238 cells were relatively resistant to growth inhibition by the HDACIs and had minimal induction of p21. Protein changes in the RAS-RAF-MEK-ERK and PI3K-AKT-mTOR pathways due to HDACIs were examined as these are important signaling proteins in thyroid cancer. Reduced levels of both pERK and pAKT were observed in all four thyroid cancer lines with both belinostat and panobinostat treatments (Fig. 1, Panel b). Also, both HDACIs caused apoptosis as measured by cleaved PARP (Fig. 1, Panel c). [No cleaved PARP was detectable in resistant T238 cultured with panobinostat 100 nM.]

**Fig. 1:** Immunoblots of thyroid cancer cell lines (BHP2-7, SW1736, T238 and Cal 62) treated with either belinostat 50 μM (Bel), panobinostat 100nM (Pan) or diluent control (Cont) (30 h) and analyzed for expression levels of various proteins. (**a**) Phosphorylated pAKT and pERK. (**b**) And cleaved PARP (*arrowhead*)

### Annexin V/propidium iodide assay

Consistent with the detection of cleaved PARP observed on Western blot, belinostat (50 μM) and panobinostat (100 nM) (30 h) induced early and late apoptosis in the BHP2-7, Cal62 and SW1736 thyroid cancer cell lines as measured by annexin V/propidium measurements (Table 2). Panobinostat (100 nM) resulted in less apoptosis (11–37 %) than belinostat (50 μM) (43–68 %). Consistent with the Western blot data, the T238 cell line had fewer apoptotic cells after culture with either panobinostat (3 %) or belinostat (24 %) as compared to the other HDACI-treated cell lines (Table 2).

**Table 2:** Annexin V/propidium iodine assay

	Control (apoptosis) (%)	Panobinostat (100 nM) (apoptosis) (%)	Belinostat (50 μM) (apoptosis) (%)
Cal62	3	37	68
SW1736	3	11	56
BHP2-7	5	16	43
T238	2	3	24

Combined early and late apoptosis results [annexin V early and propidium iodine (late) positive measured by FACS] (expressed as percentage of total number of cells) tabulated for BHP2-7, Cal62, SW1736 and T238 cell lines after 30-h culture. Results represent the mean of triplicate cultures. Means did not vary more than 10 % between experiments

### Human thyroid cancer xenograft study

Belinostat was injected intraperitoneally into immunodeficient mice carrying BHP2-7 xenografts (100 mg/kg/day, 5 days/week, 52 days). Prominent inhibition of growth of the tumors occurred in the experimental mice compared to control mice receiving diluent alone (Fig. 2a). Experimental mice did not lose body weight (Fig. 2b) and appeared and behaved normally during the study.

**Fig. 2:** Effect of belinostat on proliferation of human thyroid cancer xenografts growing in athymic mice. Graph of mean xenograft tumor volume (mm^3^) in belinostat-treated (100 mg/kg/5 day per week, I.P.) versus vehicle control-treated (treated similarly) mice over 52 days. Sixteen tumors (BHP2-7) were in both groups. (**a**) Graph of mean weights (in grams) of mice in the belinostat-treated and control-treated groups over the duration of experiment (**b**)

### TKIs and their combination with either belinostat or panobinostat with TKIs

Combinations of either belinostat or panobinostat with one of the TKIs (see Table 1) were tested against 3 thyroid cancer cell lines and assessed by MTT assay and Calcusyn^®^ analysis (Table 3a–c). HDACI–sorafenib combinations were antagonistic, while motesanib-HDACI combinations were only additive (data not shown). However, either belinostat or panobinostat with either dasatinib or pazopanib was synergistic in their anti-proliferative activity against BHP2-7 (RET/PTC rearrangement), Cal62 (KRAS mutant) and SW1736 (BRAF mutant) thyroid cancer cells. The degree of synergism varied among the above combinations but was strongest for the Cal62 cell line [i.e., combination index (CI) was lowest] (interpretation of the combination index appears on Supporting Information Fig. S1).

**Table 3:** Combination index of (a) belinostat/panobinostat and dasatinib on SW1736 cells, (b) belinostat/panobinostat and dasatinib on Cal 62 cells, (c) belinostat/panobinostat and pazopanib on BHP 2-7 cells

Dasatinib (nM)	Belinostat (nM)				Panobinostat (nM)			
(a)								
	250	500	750	1,000	1	20	40	50
100	0.47	0.41	0.39	0.29	0.14	0.48	0.54	0.56

Dasatinib (nM)	Belinostat (nM)				Panobinostat (nM)			
(b)								
	250	500	750	1,000	8	16	24	45
100	0.13	0.14	0.15	0.14	0.17	0.16	0.18	0.29

Pazopanib (μM)	Belinostat	Panobinostat
	1 μM	30 nM
1	0.66	0.50
2	0.63	0.51
3	0.52	0.47
4	0.54	–

Combination index described more fully in Fig. S1. Values ≤0.90 are consistent with synergism, and the lower the value, the greater the synergism

## Discussion

We found that belinostat and panobinostat inhibited growth in vitro, induced apoptosis and dephosphorylated AKT and ERK in a panel of thyroid cancer cell lines; and belinostat remarkably inhibited tumor growth in mice carrying thyroid cancer xenografts. Studies have shown that this family of drugs can have a myriad of effects (Dokmanovic et al. 2007). As their name implies, they can reverse the activity of HDAC, causing acetylation of histones which opens the chromatin to allow transcription of a large array of genes. Furthermore, these compounds can acetylate numerous proteins resulting in change of their function (Bolden et al. 2006). Our microarray analysis of BHP2-7 treated with either belinostat or panobinostat showed modulation of genes involved in pathways associated with the cell cycle, DNA damage and apoptosis-related processes.

The HDACIs acetylated H3 protein in the four representative cell lines, including T238 which were resistant to growth inhibition by HDACI (especially panobinostat) (Fig. 1). These cells had minimal induction of p21, suggesting that this cyclin kinase inhibitor may potentially represent a biomarker of growth inhibition by the HDACI. Various in vitro studies of MAPK and PI3K/AKT inhibitor monotherapy have shown conflicting results in thyroid cancer (depending on mutational status and growth conditions) (Schweppe et al. 2009). However, combinations of agents blocking both the PI3K-AKT-mTOR and MAPK pathways show greater anti-proliferative activity (Jin et al. 2009) and are now in clinical trials (e.g., combinations of sorafenib and everolimus) [www.clinicaltrial.gov]. We show that both belinostat and panobinostat markedly inhibited activation of both of these pathways in the four representative thyroid cancer cell lines. But T238 cells were resistant to growth inhibition by the HDACIs suggesting that inhibition of either phosphor-AKT or phosphor-ERK does not assure that the HDACI will be growth inhibitory.

One notable characteristic of thyroid cells is the ability to exchange extracellular iodine (I) for intracellular sodium (Na) by way of the Na/I symporter. The intracellular iodine has to be organified for it to stay in the cell rather than efflux out. While well-differentiated metastatic thyroid cancer can be treated with ^131^I which is selectively taken up by the thyroid Na/I symporter, radioiodine-resistant thyroid cancers are not amenable to this form of therapy. We found that belinostat and panobinostat could induce both Na/I symporter mRNA and protein in thyroid cancer cells, but the levels of intracellular ^131^I accumulation were low even though TPO was induced by these HDACIs (data not shown).

In recent years, phase II clinical trials of various small molecule tyrosine kinase inhibitors (including sorafenib, motesanib and pazopanib) (Gupta-Abramson et al. 2008; Sherman et al. 2008; Bible et al. 2010) have shown modest activity against thyroid cancers (mainly stabilization disease by RECIST criteria) (Cabanillas et al. 2010). The exact mechanism of action of these agents is still uncertain given the poor correlation between the predicted in vitro targets (e.g., RET and BRAF inhibitors) of these agents, mutational status of the tumors (RET and BRAF mutations) and clinical response. Of note, the RECIST clinical response rates of the above mentioned kinases are all remarkably similar in spite of the differences in spectrum of their kinase targets. The lack of efficacy of the tested TKIs is not surprising given our previous study (Chan et al. 2012) which showed that most thyroid cancer cell lines are either resistant to a large number of TKIs or else are effective only at high IC_50_ which are not pharmacologically relevant. A prior in vitro and in vivo study of sorafenib (Salvatore et al. 2006) showing that it was effective against a panel of BRAF V600E thyroid cancer cell lines is now known to have been confounded by the fact that most of the tested cell lines were not thyroid in origin (Schweppe et al. 2008) and that sorafenib is not a potent BRAF inhibitor.

The sensitivity of BHP2-7 (RET/PTC rearrangement) to pazopanib as well as the sensitivity of BHP2-7 and the KRAS mutant Cal62 cell line to dasatinib within the pharmacological range merits further study. The lack of efficacy of sorafenib against SW1736 (BRAF mutant) that we observed is now known to be due to the fact that sorafenib does not have potent anti-BRAF properties (Smalley and Flaherty 2009). Trials of PLX4032 in thyroid cancer, a proven potent BRAF inhibitor in melanoma, have recently been shown to have poor activity against RAS or RET mutants (Salerno et al. 2010). This is partly due to the paradoxical ability of Raf inhibitors to stimulate wild-type Raf to activate the MAPK pathway and enhance growth of these tumors (Hatzivassiliou et al. 2010).

The synergistic anti-proliferative activity of either belinostat or panobinostat combined with either pazopanib or dasatinib in the thyroid cancers carrying either RET/PTC1 rearrangement (BHP2-7), KRAS G12R mutation (Cal62) or BRAF V600E mutation (SW1736) is of interest. The mutations in these three lines are important components in the MAPK cascade. We found that the downstream pathways of these oncogenes could be inhibited by the HDACI, and thus, the TKI and HDACI may work in unison resulting in their anti-proliferative activity.

In summary, belinostat and panobinostat were effective against a wide range of thyroid cancer cell lines irrespective of their mutational composition (with the possible exception of the PI3K mutant, T238 cell line). This, in concert with the activity of belinostat to suppress the growth of thyroid cancer xenografts in athymic nude mice with no obvious side effects, suggests that clinical studies with these HDACs should be pursued. Furthermore, the synergistic combination of HDAC inhibitors-TKIs has previously not been reported and might present a clinical opportunity.

## Electronic supplementary material

Below is the link to the electronic supplementary material.

Supplementary material 1 (TIFF 116 kb)

Supplementary material 2 (TIFF 473 kb)

Supplementary material 3 (DOCX 22 kb)
